RETRACTED

# Higher Chronic Endometritis Incidences within Infertile Polycystic Ovary Syndrome Clinical Cases

**DOI:** 10.1155/2022/9748041

**Published:** 2022-04-11

**Authors:** Shuang Wang, Huishan Zhao, Fenghua Li, Yanping Xu, Hongchu Bao, Dongmei Zhao

**Affiliations:** ^1^Department of Reproductive Medicine, Qingdao University Medical College Affiliated Yantai Yuhuangding Hospital, 20 Yuhuangding East Road, Yantai 264000, China; ^2^Central Laboratory, Qingdao University Medical College Affiliated Yantai Yuhuangding Hospital, 20 Yuhuangding East Road, Yantai 264000, China

## Abstract

**Background:**

Clinical cases of a polycystic ovarian syndrome (PCOS) have prolonged subclinical inflammation. Hysteroscopy has revealed worsened chronic endometritis (CE), particularly endometrial diffuse hyperemia, in PCOS patients. However, the possible relationships between PCOS and CE remain largely unexplored.

**Methods:**

This retrospective-based investigation was conducted on 3336 infertile patients. The PCOS group consisted of 508 patients, while the non-POCS group consisted of 2828 individuals with normal ovarian function. Their clinical features and CE prevalence diagnosed with hysteroscopy were compared. The risk factors affecting the incidence of diffuse endometrial hyperemia were analyzed by binary logistic regression.

**Results:**

The PCOS cohort and the non-PCOS cohort showed marked variations in age, body mass index (BMI), infertility (primary, secondary), basal hormone level (bFSH, bLH, bT, and PRL), anti-Müllerian hormone (AMH), and CA125 (*P* < 0.05). The prevalence of CE in PCOS women was 41.73% (212/508), markedly higher than the 28.50% in the non-PCOS cohort (806/2828). Variations within diffuse endometrial hyperemia prevalence were especially marked (*P* < 0.05). Furthermore, we found that the variables of BMI, bLH, bT, and AMH correlated with diffuse endometrial hyperemia.

**Conclusions:**

CE prevalence was elevated in clinical cases of infertility associated with PCOS, and diffuse endometrial hyperemia was prevalent, as indicated by hysteroscopy. Furthermore, increased BMI, bLH, bT, and AMH levels all contribute to the risk of diffuse endometrial hyperemia.

## 1. Background

Chronic endometritis (CE) is characterized by mild endometrial inflammation. It is widely accepted that the presence of plasma cells inside the endometrial stroma is the most useful histologic criterion for diagnosis. Diagnosis of CE is often delayed, since it is usually asymptomatic [1]. Although CE does not manifest clinically, it interferes with embryo implantation and can result in reduced fertility. Recent studies have reported that the CE incidence rate is 14–42% within cases of recurring implantation failure (RIF), while this rate is 27–57.8% within cases of recurring pregnancy loss (RPL) [2]. CE is typically diagnosed through hysteroscopy and pathological examination of endometrium [3–5]. By hysteroscopy, CE is often diagnosed as micropolyps (<1 mm in size), stromal edema, or diffuse endometrial hyperemia [6, 7].

RETRACTED

Polycystic ovary syndrome (PCOS) represents a highly prevalent endocrine condition and metabolic abnormality within childbearing-aged females. It is a major cause of infertility, with the phenotypes of hyperandrogenism, insulin resistance, menstrual irregularity, hirsutism, and polycystic ovarian morphology (PCOM) [8]. In addition, PCOS patients can develop several complications, such as metabolic abnormalities, cardiovascular diseases, and psychological disorders [9]. Studies have shown that serum levels of inflammatory factors, such as interleukin 17 (IL-17), in patients with endometritis are significantly increased [10]. Furthermore, serum levels of inflammation-linked cytokines, including IL-6, C-reactive protein (CRP) and tumor necrosis factor-*α* (TNF-*α*), are increased in PCOS patients [11], and such elevation may be associated with the pathological changes in the endometrium. Currently, no data are available on the incidence of CE in PCOS patients. CE may affect the expressions of endometrial cytokines, damage the endometrial receptivity, and reduce pregnancy outcomes [12]. Moreover, CE can affect the pregnancy outcomes of infertility PCOS cases who undergo in vitro fertilization/intracytoplasmic sperm injection-embryo transfer (IVF/ICSI-ET).

This investigation retrospectively probed hysteroscopic CE clinical profiles for infertile patients with PCOS treated at our hospital.

## 2. Methods

### 2.1. Participants

Herein, a retrospective, database-searched cohort study was performed that was approved by the Yantai Yuhuangding Hospital's Institutional Review Board. Overall, 3336 infertility cases experienced hysteroscopy within the Reproductive Center of Yantai Yuhuangding Hospital from January 2018 to December 2020. Among them, 508 PCOS cases were allocated into PCOS cohort. Meanwhile, 2828 patients with normal ovarian function were allocated into non-PCOS cohort. Inclusion criteria consisted of patients diagnosed with infertility, age <40 years, and medical datasets from all cohorts compiled. Exclusion criteria were set as follows: patients with hyperprolactinemia, premature ovarian failure, and abnormal parental karyotype. The underlined diagnostic criteria for PCOS were consistent with the 2018 consensus regarding PCOS theragnostics within China [13]: spare menstruation, amenorrhea, or irregular uterine bleeding is a mandatory criterion for the diagnosis; and hyperandrogenemia or polycystic change of the ovary.

RETRACTED

### 2.2. Diagnostic Hysteroscopy of CE

The diagnosis of CE was performed with hysteroscopy. At 3–5 days after menstruation, all patients underwent gynecological examination and vaginal discharge examination to rule out contraindications for surgery, such as vaginitis and pelvic inflammatory disease. Throughout the menstrual cycle's follicular phase, all patients underwent a mini-hysteroscopic evaluation. Hysteroscopy was conducted through a lens-derived mini-telescope (Karl Storz, Tuttlingen, Germany; OD: 2.7 mm; angle vision: 105°; OD double-flow operative sheath: 4.5 mm) [14]. After disinfection of the vagina and posterior cervix, the mirror was introduced into the vagina. Subsequently, 9% sodium chloride was used to distend the uterine cavity with an expansion pressure of 100–120 mmHg. Hysteroscopy was performed using a 300 w light source through a high-definition digital-camera and a xenon bulb (Karl Storz™, Germany). Throughout this assessment, the front/rear walls, two lateral walls, both sides of the cervix, and cervical mucosa were meticulously inspected via advancing hysteroscope in-parallel across endometrial surfaces, which helped locate possible macroscopic indications of CE, including intrauterine morphology, intima color, thickness, elasticity, smoothness, glands, stroma, and fallopian tube opening [15]. This method allowed the easy detection of surface irregularities. In brief, CE was diagnosed based on the following signs: stromal edema, isolated or diffuse micropolyps, and generalized periglandular hyperemia [6, 7, 16]. The surgery for all the enrolled patients was performed by the same surgeon, which eliminated the risk of variation.

### 2.3. Ethical Consideration

The study was approved by the Yantai Yuhuangding Hospital's Institutional Review Board. All participants in this study signed a written informed consent form.

### 2.4. Statistical Analysis

All datasets were assessed through SPSS® 22.0. Continuous variables were expressed as mean ± standard deviations (SD), whereas qualitative variables reflected case quantity (*n*) together with percentages (%). Intercohort comparisons of continuous variables (normally distributed) were assessed through the dependent samples *t*-test, whereas the intercohort differences in the categorical variables (nonnormally distributed) were analyzed through contingency tables together with the chi-square test or Fisher's exact test. Logistic regression analyses probed the independent influence of multiple variables. A *P* value of <0.05 was chosen to highlight statistical significance.

RETRACTED

## 3. Results

### 3.1. Clinical Parameters

Overall, 508 cases were allocated to PCOS cohort, while 2828 cases were allocated to non-PCOS cohort.  Table 1 provides backgrounds and clinical characteristics of all cases. Considerable variations were observed regarding age, BMI, infertility (primary, or secondary), basal hormone level (bFSH, bLH, bT, and PRL), AMH, CA125, cholesterol (CHOL), and triglyceride (TG) (*P* < 0.05) across both cohorts. The BMI, the proportion of primary infertility, and the levels of bLH, bT, AMH, CHOL, and TG were all significantly higher in the PCOS cohort than in the non-PCOS cohort, but the age/bFSH, PRL, and CA125 levels were significantly lower (*P* < 0.05).

### 3.2. Prevalence of Hysteroscopic Features

Hysteroscopy demonstrated a significant increase in the diagnostic rate of CE in the PCOS cohort compared to the non-PCOS cohort (41.73% versus 28.50%) (*P* < 0.001; Figure 1).

Incidences of various hysteroscopic features associated with CE were analyzed individually. Hyperemia was detected in 24.41% of PCOS cohort cases and 8.13% of non-PCOS cohort cases, indicating that hyperemia prevalence is significantly increased in the PCOS cohort with a *P* value of <0.001 and F score of 120.276. The F-statistic is the ratio of the mean squares treatment to the mean squares error. Our obtained data revealed that most of the F values were higher, which corresponded to lower *P* values (Table 2). The prevalence of micropolyps, edema, and hyperplasia was not significantly different between the two cohorts.

### 3.3. Binary Logistic Regression Analysis: Clinical Characteristics of the Endometrial Hyperemia Cohort and Nonendometrial Hyperemia Cohort

Statistical analysis identified increased incidence rates for CE within PCOS cases, and most of them showed hysteroscopic features of endometrial hyperemia. A binary logistic regression analysis was performed to further explore associations across exposure factors and endometrial hyperemia. Clinical cases were segregated within two cohorts, depending upon endometrial hyperemia status.  Table 3 provides the background characteristics of these patients. BMI, bLH, bT, and AMH were found to be associated with endometrial hyperemia.

## 4. Discussion

For the first time, we demonstrated the common hysteroscopic characteristics linked with CE in patients with PCOS. PCOS is a multifactorial disorder of the female reproductive system that is frequently associated with metabolic disorders, such as insulin resistance, obesity, and hypertriglyceridemia [17, 18]. We found that the PCOS cohort showed higher levels of BMI (25.42 ± 3.65 vs. 23.40 ± 3.42), serum bLH (8.91 ± 4.85 vs. 5.05 ± 2.01), bT (0.40 ± 0.19 vs. 0.25 ± 0.12), AMH (0.25 ± 0.12 vs. 4.14 ± 2.67), CHOL (4.98 ± 0.94 vs, 4.74 ± 0.83), and TG (1.42 ± 0.95 vs. 1.05 ± 0.84), in comparison to the non-PCOS cohort. The findings from these datasets support previously published research. Fallopian tube blockage is the greatest driver for infertility of non-PCOS patients, which belongs to secondary infertility. Thus, age, bFSH, PRL, and CA125 levels were higher in non-PCOS cohorts compared to PCOS cohorts, indicating persistent, subclinical low-grade inflammation distinct from acute inflammation caused by bacterial or viral infections. Previous investigations demonstrated PCOS cases to have significantly upregulated chronic inflammation-linked cytokines, including IL-6, IL-8, TNF-*α*, and CRP, which may be attributed to the associated obesity, insulin resistance, and hyperandrogenemia [19, 20].

RETRACTED

At present, the CE diagnoses are defined according to endometrial biopsy findings or hysteroscopy. However, the positivity rate of endometrial biopsy is very low, at only 27.1% [21]. Hysteroscopy has been shown to increase the sensitivity/accuracy of CE diagnosis [22]. This study revealed that PCOS patients have significantly increased diagnosis rates for CE using hysteroscopy. Being a pivotal CE-diagnostic measure, hysteroscopy revealed perigonadal hyperemia, micropolyps, stromal edema, and hyperplasia within CE cases. This investigation identified CE diagnosis rate to be 41.73% within PCOS cohort, with 28.50% for non-PCOS cohort (*P* < 0.001). However, hysteroscopic features of CE in PCOS patients were slightly different in this study. Diffuse endometrial hyperemia was the most prevalent feature in the study population, showing a proportion of 24.41% and 8.13% within PCOS cohort and non-PCOS cohort, accordingly. This finding might be attributed to the increment of chronic subclinical inflammatory factors. Additionally, we found that the serum levels of bLH, bT, AMH, CHOL, and TG, as well as BMI, were markedly exacerbated within PCOS cases having CE in comparison to those with normal endometrium. Some studies have suggested that the circulatory and molecular markers of inflammation observed in CE may be associated with the circulating androgens, and the luteinizing hormone may be the progenitor of chronic inflammation [23, 24]. Hence, we hypothesized that CE in PCOS patients could be a result of a persistent inflammatory state, although the pathophysiology remains mostly unknown.

Meanwhile, we found that PCOS patients had a higher diagnosis rate of CE, and endometrial hyperemia was dominant in hysteroscopy. Accordingly, a binary logistic regression analysis was performed. Variables of BMI, bLH, bT, and AMH were related to the presence of endometrial hyperemia. Several investigations highlighted detrimental influence by obesity upon natural/assisted conception, and such a hindered reproduction ambient would be inflamed within high-BMI/central fat distribution case populations [25]. It has been reported that PCOS patients have a lower pregnancy rate than non-PCOS patients [26]. Our findings speculated that the endometrial receptivity in PCOS patients with CE was damaged. CE reflects chronic and insidious inflammatory dysfunctions within the endometrium, which triggers discharging for inflammatory mediators, congestion of the uterus, proliferation of capillaries, fibrosis, gland atrophy, and destruction of the endometrial microenvironment [27]. Pietro et al. have reported that the abnormal expressions of inflammatory response factors and apoptosis-related factors, such as IL-11, chemokine ligand 4 (CCL4), insulin-like growth factor (IGF1), B cell CLL 2 (BCL2), and BCL2-associated X protein (BAX), within CE case endometria during implantation result in decreased endometrial receptivity, resulting in embryo implantation failures [12].

RETRACTED

When evaluating this study, one of the limitations was the relatively limited sample size, as large sample sizes are required for retrospective studies. Additionally, the retrospective aspect may introduce selection bias, which should be considered.

## 5. Conclusion

In conclusion, CE incidence rates were significantly increased in PCOS patients, and endometrial hyperemia was the most common hysteroscopic finding in CE patients. For the first time, we showed the relationship between endometrial hyperemia and PCOS. Within this univariate analysis, BMI, bLH, bT, and AMH were the risk factors leading to endometrial hyperemia. Moreover, further investigations are needed to explore the mechanisms underlying these effects.

## Figures and Tables

**Figure 1:** Different features of chronic endometritis at fluid hysteroscopy: (a) diffuse hyperemia endometrium, (b) micropolyps (less than 1 mm in size), and (c) edema hyperplasia.

**Table 1:** Clinical characteristics of patients (PCOS and non-PCOS cohorts).

	PCOS cohort (*n* = 508)	Non-PCOS cohort (*n* = 2828)	*P* value
Age, years	31.03 ± 3.20	31.98 ± 3.57	<0.001
Infertility duration, years	3.86 ± 2.32	3.65 ± 2.35	0.056
BMI (kg/m^2^)	25.42 ± 3.65	23.40 ± 3.42	<0.001
Infertility			
Primary infertility %	280 (55.12%)	1410 (49.86%)	0.029
Secondary infertility %	228 (44.88%)	1418 (50.14%)	
bFSH (UI/L)	5.94 ± 1.41	6.84 ± 1.89	<0.001
bLH (UI/L)	8.91 ± 4.85	5.05 ± 2.01	<0.001
bE_2_ (pg/ml)	35.45 ± 12.01	34.43 ± 13.86	0.128
bP (ng/ml)	0.50 ± 0.30	0.52 ± 0.25	0.055
bT (ng/ml)	0.40 ± 0.19	0.25 ± 0.12	<0.001
PRL (ng/ml)	16.30 ± 6.55	17.35 ± 6.13	0.001
AMH (ng/ml)	10.08 ± 6.36	4.14 ± 2.67	<0.001
CA125 (U/ml)	16.98 ± 7.88	23.87 ± 9.59	<0.001
CHOL (mmol/L)	4.98 ± 0.94	4.74 ± 0.83	<0.001
LDL-C (mmol/L)	2.98 ± 0.81	2.81 ± 0.67	0.241
TG (mmol/L)	1.42 ± 0.95	1.05 ± 0.84	<0.001

bFSH, basal follicle-stimulating hormone; bLH, basal luteinizing hormone; bE_2_, basal estradiol; bP, basal progesterone; bT, basal total testosterone; PRL, prolactin. The limit of significance is a *P* value <0.05, which was evaluated on the basis of the chi-square test.

RETRACTED

**Table 2:** Hysteroscopic features in the PCOS and non-PCOS cohorts.

	PCOS cohort (*n* = 508)	Non-PCOS cohort (*n* = 2828)	*F*	*P* value
CE	212 (41.73%)	806 (28.50%)	35.557	<0.001
Hyperemic %	124 (24.41%)	230 (8.13%)	120.276	<0.001
Micropolyps %	15 (2.95%)	118 (4.17%)	1.674	0.196
Edema hyperplasia %	73 (14.37%)	458 (16.20%)	1.072	0.301
Normal %	258 (50.79%)	1656 (58.56%)	10.631	<0.001
Endometrial macropolyps %	31 (6.10%)	234 (8.27%)	2.778	0.096
Others	7 (1.38%)	132 (4.67%)	11.671	<0.001

Others are intrauterine adhesions, uterine malformations, submucosal fibroids of the uterus, and endometrium atypical hyperplasia.

**Table 3:** Clinical characteristics of endometrial hyperemia and nonendometrial hyperemia cohorts.

	Hyperemia cohort (*n* = 354)	Nonhyperemia cohort (*n* = 2982)	*P* value	95% CI
Age, years	31.19 ± 3.52	31.89 ± 3.52	0.101	0.925–1.007
Infertility duration, years	3.80 ± 2.37	3.75 ± 2.52	0.792	0.950–1.070
BMI (kg/m^2^)	24.77 ± 3.39	23.64 ± 3.46	<0.001	1.064–1.164
Infertility				
Primary infertility %	192 (54.24%)	1498 (50.23%)	0.855	0.775–1.235
Secondary infertility %	162 (45.76%)	1484 (49.77%)		
bFSH (UI/L)	6.53 ± 1.77	6.71 ± 1.87	0.975	0.914–1.097
bLH (UI/L)	6.91 ± 4.10	5.57 ± 3.01	<0.001	1.058–1.149
bE_2_ (pg/ml)	34.33 ± 13.78	34.77 ± 13.94	0.774	0.998–1.009
bP (ng/ml)	0.50 ± 0.29	0.52 ± 0.26	0.144	0.380–1.152
bT(ng/ml)	0.32 ± 0.16	0.26 ± 0.14	<0.001	4.917–19.946
PRL (ng/ml)	16.74 ± 6.59	17.30 ± 6.25	0.823	0.976–1.019
AMH (ng/ml)	7.21 ± 4.83	4.92 ± 2.78	<0.001	1.028–1.095
CA125 (U/ml)	20.89 ± 8.85	22.99 ± 7.17	0.470	0.997–1.007
CHOL(mmol/L)	4.83 ± 0.87	4.78 ± 0.86	0.880	0.559–1.647
LDL-C (mmol/L)	2.84 ± 0.78	2.85 ± 0.95	0.946	0.558–1.724
TG (mmol/L)	1.22 ± 0.92	1.08 ± 0.86	0.675	0.731–1.225

## Data Availability

The data used to support the findings of this study are available from the corresponding author upon request.

## Abbreviations

PCOS: Polycystic ovary syndrome
CE: Chronic endometritis
IVF: In vitro fertilization
RIF: Recurrent implantation failure
RPL: Recurrent pregnancy losses
AMH: Anti-Müllerian hormone
T: Testosterone.
